The article "KCNQ1OT1 Influences HK-2 Apoptosis and Inflammation in LPS-Induced Acute Renal Injury via Modulating miR-30a-5p/NLRP3 Axis" was retracted in 2023. Reasons: signs of a paper mill; suspected computer-generated content; unreliable results or conclusions; concerns about the data.

# KCNQ1OT1 Influences HK-2 Apoptosis and Inflammation in LPS-Induced Acute Renal Injury via Modulating miR-30a-5p/NLRP3 Axis

**DOI:** 10.1155/2022/2789900

**Published:** 2022-12-06

**Authors:** Jing Hou, Jun-Ming Fan

**Affiliations:** ^1^Department of Geriatrics, The Affiliated Hospital of Southwest Medical University, Luzhou, China; ^2^Chengdu Medical College Southwest Medical University, Chengdu, China

## Abstract

**Objective:**

To investigate the influence of KCNQ1OT1 on HK-2 apoptosis and inflammation in ARI and its molecular mechanism.

**Methods:**

Normal cultivated HK-2 cells were used as negative control (NC) group. Three different concentrations of lipopolysaccharide (LPS) were used to treat the cells (5 *μ*g/mL, 10 *μ*g/mL, and 20 *μ*g/mL). The groups included si-KCN1OT1+ LPS, si-NC + LPS, miR-30a-5p + LPS, pcDNA-NLRP3+si-KCNQ1OT1 + LPS group, miR-NC + LPS group, and pcDNA + si-KCNQ1OT1 + LPS group. CCK-8 and flow cytometry are used to measure cell viability and apoptosis, while RT-qPCR and Western blotting are used to detect KCNQ1OT1, miR-30a-5p, and NLRP3 mRNA. ELISA was used to detect the levels of TNF-*α*, IL-6, and IL-1*β* in HK-2 cells. The targeting relationship among KCNQ1OT1, miR-30a-5p, and NLRP3 was verified.

**Results:**

After the intervention of LPS, the viability of HK-2 cells was decreased, while the apoptosis rates were increased. The mRNA and protein expressions of NLRP3 and KCNQ1OT1 were increased, while the mRNA and protein levels of miR-30a-5p were decreased (*P* < 0.05). The expressions of Bax and Cleaved-caspase-3 were downregulated after silencing KCNQ1OT1 and overexpressed miR-30a-5p. In addition, the viability of HK-2 cells was improved, and the apoptosis was reduced by inhibiting KCNQ1OT1 and overexpressed miR-30a-5p. Thus, KCNQ1OT1 modulated NLRP3 via targeting miR-30a-5p. Overexpression of NLRP3 reverses KCNQ1OT1 inhibition of LPS-induced apoptosis, activity, and inflammation in HK-2 cells.

**Conclusions:**

Through modulating the miR-30a-5p/NLRP3 axis, inhibition of KCNQ1OT1 may reduce HK-2 apoptosis and inflammation in LPS-induced ARI.

## 1. Introduction

ARI (acute renal injury) is a pathology caused by thrombosis in the renal organ, which can easily lead to occlusion or even renal necrosis and seriously endangers normal renal function. However, acute respiratory infection is a rare disease that does not have authoritative material or medical reports to confirm its incidence. Different doctors and scholars also hold different research views on ARI. Although the incidence of ARI is low, it is easy to be misdiagnosed by doctors, and misdiagnosis of ARI brings irreversible physical damage to patients. ARI is a clinical syndrome caused by a rapid decline in renal function due to various causes. RTEC (renal tubular epithelial cell) injury is the central link causing ARI. Besides, oxidative stress (OS) injury and renal tissue inflammation are also related to its pathological mechanism. Therefore, understanding the relevant pathogenic mechanism can provide a reference for targeted therapy research [1,2]. NLRP3 inflammasomes are important proteins that mediate the body's innate immune response, regulating the inflammatory response by mediating the maturation and release of various pro-inflammatory factors. Relevant research has shown that inflammasome-dependent and inflammasome-independent NLRP3 can interfere with the progression of renal diseases by regulating inflammatory responses and apoptosis of RTECs [3,4]. NLRP3 inflammasome activation can promote sepsis-induced ARI [5,6]. At the same time, inhibition of NLRP3 inflammasome can attenuate apoptosis in contrast to agent-induced ARI by upregulating HIF1A and BNIP3-mediated mitochondrial autophagy [7].

miRNAs are potential biomarkers for detecting kidney and other organ damage. In this study, the miRNAs that can regulate NLRP3 were predicted by biological software, and NLRP3 was found to have binding loci with miR-30a-5p. Moreover, miR-30a-5p is significantly aberrant in patients with severe ARI [8,9]. Besides, lncRNA H19 overexpression alleviates ischemic ARI through miR-30a-5p [10]. However, the mechanism of miR-30a-5p′s impact on apoptosis and inflammatory response of HK-2 cells in ARI remains unclear. Potassium voltage-gated channel, KQT-like subfamily, and KCNQ1OT1, a lncRNA found at the KCNQ1 locus, have binding loci with miR-30a-5p. It is reported that interference with KCNQ1OT1 can reduce high glucose-induced HK-2 inflammation, pyroptosis, and OS [11]. In addition, KCNQ1OT1 can promote the pyroptosis of podocytes under SC5B-9 inducement by upregulating NLRP3 and suppressing miR-486a-3p [8]. However, it remains unclear whether the mechanism of KCNQ1OT1 on apoptosis and inflammation of HK-2 in ARI is associated with miR-30a-5p and NLRP3. Accordingly, an ARI model was built by intervening HK-2 with lipopolysaccharide (LPS) to investigate whether KCNQ1OT1 could influence LPS-induced HK-2 apoptosis and inflammatory action via modulating miR-30a-5p/NLRP3.

## 2. Materials and Methods

### 2.1. Materials

HK-2 (Newgain Biotech, Wuxi, CHN); RPMI-1640 culture medium (Yipu Biology, Wuhan, CHN); LPS, Trizol reagent and RIPA protein lysate (Biolab Biotech, Beijing, CHN); CCK-8 and apoptosis detection kits (Jingkehuaxue, Shanghai, CHN); reverse transcription kit and fluorescence quantitative PCR kit (Zhennuo Biotech, Shanghai, CHN); IL-1*β*, TNF-*α*, and IL-6 ELISA kits (Caiyou Industrial, Shanghai, CHN); dual luciferase reporter gene detection kit (Amyjet Scientific, Wuhan, CHN).

### 2.2. Cell Processing and Grouping

RTECs are usually cultured with RPMI-1640 medium and treated with 5.0, 10.0, and 20.0 *μ*g/mL LPS, respectively, as LPS groups with different concentrations, among which 20.0 *μ*g/mL LPS treated group was the LPS group. Normal cultivated cells were used as negative control (NC) group.

KCNQ1OT1 small interfering (si) RNA expression vector and NC as well as miR-30a-5p mimics and NC were transfected into HK-2, respectively. Subsequently, it was intervened by LPS (20.0 *μ*g/mL) and assigned to si-KCNQ1OT1+LPS group, si-NC + LPS group, miR-30a-5p + LPS group, and miR-NC + LPS group, respectively. NLRP3 overexpression vector and NC were co-transfected into HK-2, respectively, and then it was intervened by LPS at 20.0 *μ*g/mL, as pcDNA-NLRP3+si-KCNQ1OT1+LPS group and pcDNA + si-KCNQ1OT1+LPS group.

### 2.3. CCK-8

Cells were inoculated in the 96-well plates for 24 h and then treated with a CCK-8 reagent (10 *μ*L) for 2 h. The absorbance value (A; 450 nm) was calculated with a microplate reader.

### 2.4. Apoptosis Determined by Flow Cytometry (FCM)

After 48 h of culture, the cells were subjected to two precooled PBS rinses and mixed with 500 *μ*L binding buffer. Then, they were put into Annexin V-FITC (10 *μ*L) and PI (5 *μ*L) and cultivated for 10 min away from light after thorough mixing. Becton Dickinson Calibur detected apoptosis rate.

### 2.5. RT-qPCR

The total RNA of each group was isolated and reverse transcribed to cDNA for PCR. The relative expression relative to *β*-actin and U6 was calculated by the 2^−△△Ct^ method (see Table 1 for details).

### 2.6. Western Blot

Total proteins were extracted from HK-2 cells, and the protein concentrations were detected by BCA working reagent. Then, the proteins were electrically transferred to polyvinylidene fluoride (PVDF) membranes. PVDF membranes were blocked with nonfat-dried milk (5%, indoor temperature) for 1 h and cultivated overnight (4°C) with primary antibodies of NLRP3, Bax, and Cleaved-caspase-3 (1 : 1000). Then, it was immersed with the secondary antibody (1 : 2,000) for two hours at ambient temperature. ECL reagents are used for imaging, and the gray levels of proteins were analyzed with Quantity One.

### 2.7. ELISA

After 48 h of culture, carefully collect the supernatant of cells in each set of dishes and operate according to the instructions of the kit. Finally, blank wells were zeroed, and OD_450nm_ was measured with a microplate analyzer. A standard curve (abscissa: the standard substance's concentration, ordinate: OD value) was drawn, and the corresponding concentration was found from the standard curve based on the sample's OD value.

### 2.8. Dual-Luciferase

Two gene vectors were established, KCNQ1OT1 and NLRP3, respectively, incorporating miR-30a-5p. Also, miR-NC was selected for co-transfection into HK-2, and miR-30a-5p was also selected. Activity detection is based on corresponding specifications and instructions. Si-KCNQ1OT1 and si-NC were transfected into HK-2 cells, and then si-KCNQ1OT1 was co-transfected into HK-2 cells after being transfected with miR-30a-5p inhibitor and si-NC. RT-qPCR measured the miR-30a-5p level, and the protein expressions of NLRP3 were tested by WB.

### 2.9. Statistical Analysis

SPSS 20.0 was used for date analysis. The data were represented as mean ± standardization (*x* ± *s*). Two independent samples were identified by *T* test, and one-way ANOVA was used for multiple groups. The difference had statistical significance (*P* < 0.05).

## 3. Results

### 3.1. Impacts of Different Concentrations of LPS on HK-2 Activity and Apoptosis

The activity and apoptosis of HK-2 cells at different LPS (5, 10, and 20 *μ*g/mL) concentrations were detected. CCK-8 and FCM were used to measure the current activity coefficient and death percentage of HK-2 cells, respectively. The data of the two methods suggest that with the increase of LPS concentration, the activity gradually decreases and mortality gradually increases (*P* < 0.05, as shown in Figure 1). The results showed that LPS inhibited the activity of HK-2 cells and that high concentrations of LPS were closely associated with cell death.

### 3.2. Impacts of LPS at Different Concentrations on KCNQ1OT1, miR-30a-5p, and NLRP3

HK-2 was treated with different concentrations of LPS (5, 10, 20 *μ*g/mL), and the expression of KCNQ1OT1, miR-30a-5p and NLRP3, and NLRP3 protein in cells at different LPS concentrations were detected by RT-qPCR and WB, respectively. As shown in Figure 2, as the LPS concentration increased, KCNQ1OT1 showed a common increase trend, and miR-30a-5p changed in the opposite direction, decreasing. Also, the expression of NLRP3 mRNA and protein increased, and there is also a dose-dependent characteristic (*P*<0.05). LPS can increase the expression levels of KCNQ1OT1 and NLRP3, but a drop follows miR-30a-5p.

### 3.3. Impacts of si-KCNQ1OT1 on Activity, Apoptosis, and Inflammation (TNF-*α*, IL-6, and IL-1*β*) of HK-2 under LPS Induction

When transfected with si-NC and si-KCNQ1OT1, the cells were treated with LPS at a concentration of 20.0 *μ*g/mL. The expression of KCNQ1OT1 was detected by RT-QPCR, the protein expression of Bax was detected by WB, and the level of TNF-*α* etc. was detected by ELISA. In addition, cell activity was determined by CCK-8 assay, and FCM detected cell apoptosis rate. LPS group showed elevated KCNQ1OT1, Cleaved-caspase-3, and Bax, decreased HK-2 activity, enhanced apoptosis, and increased inflammatory cytokines than NC. Compared with the si-NC + LPS group, KCNQ1OT1, Bax, and Cleaved-caspase-3 reduced in the si-KCNQ1OT1+LPS group, HK-2 activity increased, apoptosis rate decreased, and IL-1*β*, TNF-*α*, and IL-6 decreased (*P* < 0.05, Figure 3). The results showed that downregulating KCNQ1OT1 inhibited LPS-induced apoptosis and produced si-KCNQ1OT1 to affect activity, apoptosis, and inflammation.

### 3.4. Overexpression Impacts

HK-2 cells were treated with 20.0 *μ*g/mL LPS after transfection of miR-NC. ELISA detected the expressions of TNF-*α*, IL-6, and IL-1*β*. FCM measured the apoptosis rates, and the protein levels of Bax and Cleaved-caspase-3 were tested by WB. It indicates that miR-30a-5p is increased, the activity of HK-2 increased, the levels of TNF-*α*, IL-6, and IL-1*β* decreased, the apoptosis rate decreased, and Bax and Cleaved-caspase-3 decreased in miR-30a-5p + LPS (Figure 4). It indicates that when overexpression occurred, LPS-induced HK-2 mortality was controlled, and inflammation was alleviated.

### 3.5. KCNQ1OT1 Regulates NLRP3 Expression via Targeting miR-30a-5p

LncBase Predicted v.2 predicted that KCNQ1OT1 had binding loci with miR-30a-5p (Figure 5(a)). Also, TargetScan prediction revealed that miR-30a-5p and NLRP3 had binding loci (Figure 5(b). According to the genetic test report, in the test cells, the activity of the luciferase substance decreased after co-transfecting miR-30a-5p with KCNQ1OT1 and NLRP3 wild-type reporter plasmids (*P* < 0.05, Figures 5(c) and 5(d)). After downregulating KCNQ1OT1 alone and simultaneously downregulating KCNQ1OT1 and miR-30a-5p, expression of the latter in HK-2 cells was detected by RT-qPCR, and WB detected the protein expression of NLRP3. It was found that miR-30a-5p in si-KCNQ1OT1 increased and NLRP3 decreased. The miR-30a-5p was decreased in the si-KCNQ1OT1+anti-miR-NC group compared with the si-KCNQ1OT1+anti-miR-30a-5p group, while NLR3 was increased. The miR-30a-5p was decreased in the si-KCNQ1OT1+anti-miR-NC group and increased in the NLR3 compared to the si-KCNQ1OT1+anti-miR-30a-5p group.

### 3.6. NLRP3 Overexpression Can Reverse si-KCNQ1OT1's Effect on Viability, Apoptosis, and Inflammatory Reaction of HK-2 under LPS Induction

The results showed that compared with pcDNA + si-KCNQ1OT1+LPS group, NLRP3, Bax, and Cleaved-caspase-3 increased in pcDNA-NLRP3+si-KCNQ1OT1+LPS group, HK-2 cell activity decreased, apoptosis enhanced, and IL-1*β*, TNF-*α*, and IL-6 contents increased (*P* < 0.05, Figure 6). It shows that NLRP3 overexpression can attenuate the effect of downregulating KCNQ1OT1 on LPS-induced HK-2 cell activity, apoptosis, and inflammation.

## 4. Discussion

In conclusion, this study found that inhibition of KCNQ1OT1 reduced HK-2 LPS-induced apoptosis and inflammatory responses in ARI cells by modulating the miR-30a-5p/NLRP3 axis (Figure 7).

ARI is a common and serious clinical condition [12,13]. RTEC injury and the resulting inflammatory reaction are important pathophysiological mechanisms of ARI, so inhibiting RTEC injury and inflammatory reaction is one of the important means to prevent and treat ARI [14,15]. It has been reported that ncRNAs of lncRNAs and miRNAs are essential in kidney injury and repair and play important roles as biomarkers and therapeutic targets of ARI [16]. KCNQ1OT1 can upregulate Tead1 to induce cardiomyocyte apoptosis in the acute myocardial infarction model [17]. In addition, LPS-induced increase in KCNQ1OT1 in HMC3 cells and inhibiting KCNQ1OT1 can reduce LPS-induced neuroinflammation and neuron apoptosis through modulating miR-30e-3p/NLRP3 [18–21]. Knocking down KCNQ1OT1 is shown to significantly alleviate the inflammation, OS, and apoptosis of PC12 under the inducement of oxygen-glucose deprivation and reperfusion [22,23]. The results of this study identified elevated KCNQ1OT1 in HK-2 under LPS inducement. Inhibiting KCNQ1OT1 gave rise to reduced Bax and Cleaved-caspase-3 expression, enhanced HK-2 activity, decreased apoptosis, and reduced IL-1*β*, TNF-*α*, and IL-6 contents. It suggests that inhibition of KCNQ1OT1 can reduce apoptosis and inflammation of LPS-induced HK-2 cells, which is similar to previous studies, indicating that KCNQ1OT1 has anti-inflammatory and anti-injury effects.

A study has reported that via targeting GLUD1, miR-30a-5p inhibits OS and apoptosis of RTEC HK-2 under hypoxia/reoxygenation inducement [24,25]. Besides, miR-30a-5p can relieve inflammatory damaged A549 and mice induced by LPS [26] by targeting RUNX2. Also, upregulating miR-30a-5p is capable of promoting the growth of immortalized rat podocyte lines and inhibiting its apoptosis, thus ameliorating the podocyte defects caused in vitro [27]. This paper unveiled decreased miR-30a-5p in HK-2 induced by LPS. Overexpressing miR-30a-5p decreased Cleaved-caspase-3, Bax, and inflammatory cytokines, enhanced HK-2 activity, and reduced apoptosis. Overexpressing miR-30a-5p could inhibit apoptosis and inflammation of HK-2 under LPS inducement. In addition, this experiment found that KCNQ1OT1 can regulate miR-30a-5p expression, suggesting that KCNQ1OT1 may influence apoptosis and inflammation of HK-2 under LPS inducement by modulating miR-30a-5p.

Harmine can alleviate LPS-induced ARI by inhibiting the TLR4-NF-kappaB/NLRP3 inflammasome axis [5,28]. LncRNA ANRIL promotes NLRP3 inflammasome excitation through upregulation of BRCC3 [29]. The above studies indicate that NLRP3 relates to ARI and the resulting inflammatory reaction. Overall, this research found that NLRP3 mRNA and protein increased in HK-2 under LPS inducement, which indicated that NLRP3 might be activated in HK-2 injured by LPS. In addition, miR-30a-5p can bind to NLRP3 targeting, and KCNQ1OT1 can regulate NLRP3 by targeting miR-30a-5p. Moreover, overexpressing NLRP3 can reverse the influence on activity.

To sum up, through the modulation of miR-30a-5p/NLRP3, inhibiting KCNQ1OT1 may suppress apoptosis and inflammation of HK-2 in LPS-induced ARI.

## Figures and Tables

**Figure 1:** Effects of different concentrations of LPS on HK-2 viability and apoptosis. (a) Cell proliferation detected by CCK-8. (b) Histogram of apoptosis rate. (c) Apoptosis detected by flow cytometry. Note: ^*∗*^*P* < 0.05 vs NC.

**Figure 2:** Effects of LPS at different concentrations on the expression of KCNQ1OT1, miR-30a-5p, and NLRP3 in HK-2 cells. (a) KCNQ1OT1 expression in HK-2 cells detected by RT-qPCR. (b) miR-30a-5p expression in HK-2 cells detected by RT-qPCR. (c) NLRP3 mRNA expression in HK-2 cells detected by RT-qPCR. (d) NLRP3 protein expression in HK-2 cells detected by Western blot. Note: ^*∗*^*P* < 0.05 vs NC.

**Figure 3:** Effects of si-KCNQ1OT1 on LPS-induced HK-2 cell viability, apoptosis, and inflammation. (a) KCNQ1OT1 expression in HK-2 cells detected by RT-qPCR. (b) Cell proliferation determined by CCK-8. (c) Changes in the expression of inflammatory cytokines. (d) Apoptosis measured by flow cytometry. (e) Bax and Cleaved-caspase-3 protein expression detected by Western blot. Note: ^*∗*^*P* < 0.05 vs NC; #*P* < 0.05 vs si-NC + LPS.

**Figure 4:** Effects of overexpression of miR-30a-5p on LPS-induced HK-2 cell viability, apoptosis, and inflammatory response. (a) miR-30a-5p expression in HK-2 cells detected by RT-qPCR. (b) Cell proliferation determined by CCK-8. (c) Changes in the expression of inflammatory cytokines. (d) Cell apoptosis determined by flow cytometry. (e) Bax and Cleaved-caspase-3 protein expression detected by Western blot. Note: ^*∗*^*P* < 0.05 vs miR-NC + LPS.

**Figure 5:** KCNQ1OT1 regulates the expression of NLRP3 by targeting miR-30a-5p. (a) The binding sites of KCNQ1OT1 and miR-30a-5p predicted by LncBase Predicted v.2. (b) The binding sites of miR-30a-5p and NLRP3 predicted by TargetScan. (c) Detection of luciferase activity after co-transfection of miR-NC or miR-30a-5p and KCNQ1OT1 reporter plasmid into HK-2 cells. (d) Detection of luciferase activity after co-transfection of miR-NC or miR-30a-5p and NLRP3 reporter plasmid into HK-2 cells. (e) miR-30a-5p expression in HK-2 cells detected by RT-qPCR. (f) NLRP3 expression detected by Western blot.

**Figure 6:** NLRP3 overexpression can reverse the effect of si-KCNQ1OT1 on LPS-induced HK-2 cell viability, apoptosis, and inflammatory reaction. (a) Cell proliferation detected by CCK-8. (b) Changes in the expression of inflammatory cytokines. (c) Apoptosis determined by flow cytometry. (d) NLRP3, Bax, and Cleaved-caspase-3 protein expression detected by Western blot. Note: ^*∗*^*P* < 0.05 vs pcDNA + si-KCNQ1OT1+LPS group.

**Figure 7:** The mechanism of KCNQ1OT1 influences HK-2 apoptosis and inflammation in LPS-induced acute renal injury.

**Table 1:** Primer sequences.

Gene	Upstream	Downstream
KCNQ1OT1	5′-CTTTGCAGCAACCTCCTTGT-3′	5′-TGGGGTGAGGGATCTGAA-3′
NLRP3	5′-CCCCGTGAGTCCCATTA-3′	5′-GACGCCCAGTCCAACAT-3′
*β*-Actin	5′-GAGCTACGAGCTGCCTGACG-3′	5′-GTAGTTTGGTGGATGCCACAG-3′
miR-30a-5p	5′-GGGCCTGTAAACATCCTCG-3′	5′-GAATACCTCGGACCCTGC-3′
U6	5′-GGTCGGGCAGGAAAGAGGGC-3′	5′-GCTAATCTTCTCTGTATCGTTCC-3′

## Data Availability

The datasets used and analyzed during the current study are available from the corresponding author upon reasonable request.
